# *MiR-29a*: a potential therapeutic target and promising biomarker in tumors

**DOI:** 10.1042/BSR20171265

**Published:** 2018-02-08

**Authors:** Jin-yan Wang, Qian Zhang, Dan-dan Wang, Wei Yan, Huan-huan Sha, Jian-hua Zhao, Su-jin Yang, He-da Zhang, Jun-chen Hou, Han-zi Xu, Yun-jie He, Jia-hua Hu, Shan-liang Zhong, Jin-hai Tang

**Affiliations:** 1 Department of General Surgery, The Affiliated Cancer Hospital of Nanjing Medical University & Jiangsu Cancer Hospital & Jiangsu Institute of Cancer Research, Nanjing 210009, P.R. China; 2 The Fourth Clinical School, Nanjing Medical University, Nanjing 210029, P.R. China; 3 Center of Clinical Laboratory Science, Jiangsu Cancer Hospital & Jiangsu Institute of Cancer Research & The Affiliated Cancer Hospital of Nanjing Medical University, Nanjing 210009, P.R. China; 4 Department of General Surgery, Southeast University Medical School, Nanjing, Jiangsu, P.R. China; 5 Department of Radiation Oncology, Jiangsu Cancer Hospital, Nanjing, Jiangsu, P.R. China; 6 Department of General Surgery, The First Affiliated Hospital of Nanjing Medical University, Nanjing 210029, P.R. China

**Keywords:** biomarkers, cancer, metastases, microRNA, miR-29a, proliferation

## Abstract

MiRNAs, small non-coding RNA molecules, were recognized to be associated with the incidence and development of diverse neoplasms. MiRNAs were small non-coding RNAs that could regulate post-transcriptional level by binding to 3′-UTR of target mRNAs. Amongst which, *miR-29a* was demonstrated that it had significant impact on oncogenicity in various neoplasms through binding to critical genes which enhanced or inhibited the progression of cancers. *MiR-29a* participated in kinds of physiological and pathological processes, including virus replication, cell proliferation, differentiation, apoptosis, fibrosis, angiogenesis, tumorigenicity, metastasis, drug-resistance, and so on. According to its sufficient sensitivity and specificity, many studies showed that *miR-29a* might serve as a potential therapeutic target and promising biomarker in various tumors. In this review, we discussed the functions of *miR-29a* and its potential application in the diagnosis, treatment and stages of carcinoma, which could provide additional insight to develop a novel therapeutic strategy.

## Introduction

Mortality caused by cancer is soaring globally, which urgently requests us to figure out a safe and effective way to further improve overall survival of tumor patients [1]. Then, molecular targetting treatment of cancer entered our sight and brought cancer patients a ray of dawn. Based on massive researches, miRNAs appeared to modulate various pathways in malignant neoplasms, which might offer a brand new and effective way in future molecular targetting cancer treatment [2,3]. MiRNAs are a class of small, highly conserved, time sequencing, and non-coding RNAs, including 18–25 nts, that regulate gene expression at both transcriptional and post-transcriptional levels. They are involved in different biological and metabolic processes, through binding to the 3′-UTRs of mRNAs [4]. Additionally, miRNAs are disclosed that they are related to many biological processes including cell proliferation, apoptosis, angiogenesis, drug-resistance, invasion, and metastasis [5]. Cho [6] had summarized miRNAs as a potential biomarker for diagnosis, prognosis, and therapy with ample evidence in cancers. Liu et al. [7] highlighted multifarious miRNAs participated in the regulation of chemoresistance, cell cycle, and apoptosis in the process of epithelial-to-mesenchymal transition (EMT), cell cycle, and apoptosis in colorectal cancer (CRC) cells. For instance, *miR-139-5p* inhibited cell proliferation of breast cancer (BCa) [8]. *MiR-335* promoted gastric cancer (GC) cell apoptosis by targetting CT10 oncogene homolog-like (CRKL) [9]. *MiR-222* mediated adriamycin resistance to BCa cells [10]. *MiR-22* decreased migration due to down-regulating CD147 expression in tongue squamous cell carcinoma (TSCC) [11].

*MiR-29* family (*miR-29a, miR-29b*, and *miR-29c*) was connected with aggressiveness and prognosis of malignant neoplasms and might act as a considerable biomarker for forecasting the recurrence and progression of cancers [12–15]. Nonetheless, from articles we have learnt that *miR-29a* and *miR-29b* appeared to be more effective than *miR-29c* in targetting genes and signaling pathways [16,17]. The role of *miR-29b* in cancers had been fully discussed by Yan et al. [18] in 2015 and the new progression of *miR-29b* was less. Yet, the function of *miR-29a* had not been sufficiently summarized. On account of available researches, *miR-29a* had been found to be associated with kinds of neoplasms. For instance, it was down-regulated in metastatic prostate cancer (PCa) [19], myeloid leukemias [20], endocrine-sensitive BCa [21], lung cancer [22], ALK-positive anaplastic large cell lymphomas (ALCLs) [23], oral squamous carcinoma (OSCC) [24], glioblastoma [25]. Interestingly, other findings proclaimed that *miR-29a* was up-regulated in cholangiocarcinoma [26], CRC [27], and so on. Apart from its role in cancer, miRNAs were also involved in a variety of non-malignant diseases. According to Wei et al. [28], miRNAs served as a potential biological role in the initiation of pulmonary inflammation. Without exception, *miR-29a* was correlated with kinds of non-malignant diseases, like Alzheimer’s disease [29], cholestatic pediatric liver disease [30], atherosclerosis [31], atrial fibrillation [32], active pulmonary tuberculosis [33], thoracic aneurysms [34], tendon disease [35], hepatic fibrosis [36], ankylosing spondylitis [37], diabetes [38], scleroderma [39], and fatty liver disease [40]. Besides, evidence had proved that *miR-29a* greatly participated in multifarious cell processes, such as cell proliferation, apoptosis, angiogenesis, invasion, and metastasis and drug-resistance [41–43]. Thus it could been seen that *miR-29a* might play a considerable role in the adjustment of kinds of diseases, especially cancers. In this review, we will focus on the action of *miR-29a* in the processes of cell proliferation, apoptosis, angiogenesis, invasion, metastasis, and drug resistance, and work out the network of genes modulating its functions, and predict the potential role of *miR-29a* in the diagnosis and molecular targetted therapy of human cancers.

### *MiR-29a* in cell proliferation

An increasing number of studies showed that *miR-29a* was correlated with proliferation to a great extent. TUT1, a nucleotidyl transferase, could increase the expression of *miR-29a*, then inhibiting PPARγ and SREBP-1c expression, which suppressed cell proliferation in osteosarcoma (OS) [44]. Li et al. [41] discovered that *miR-29a* repressed PCa cell proliferation and development of PCa through targetting lysine demethylation 5B (KDM5B). KDM5B could specifically reduce the methylation levels of histone H3 at lysine 4 (H3K4). Additionally, Cui et al. [45] confirmed that, in GC, *miR-29a* could suppress the expression level of p42.3 which had been proved to be associated with cell proliferation. Consequently, *miR-29a* might act as an inhibitor in the modulation of cell proliferation. Lately, Zhao et al. [46] also found that, *in vitro*, enhancing the expression of *miR-29a* could decrease cell proliferation in GC via diluting the level of Cyclin-dependent kinase (CDK) 2 (CDK2), CDK4, and CDK6. Furthermore, cell proliferation could also be directly refrained by *miR-29a* through suppressing the expression of Mucin 1 (MUC1). MUC1 was a membrane-bound glycoprotein, interacting with the epidermal growth factor receptor (EGFR) [47]. Besides, MUC1, targetted by *miR-29a*, was also lately confirmed to accommodate in pancreatic ductal adenocarcinoma (PDAC) cell proliferation through p42-44 MAPK and β-catenin pathways [48]. Moreover, according to Xi et al. [25], *miR-29a* repressed the level of Wilms’ tumor 1-associating protein (WTAP), phosphoinositide 3-kinase (PI3K)/protein kinase B (PKB)/AKT and extracellular signal-related kinase pathways through targetting Quaking gene isoform 6 (QKI-6) in glioblastoma stem cells (GSCs), accordingly inhibiting cell proliferation. Zhu et al. [49] recognized that osteonectin (SPARC) restrain the phosphorylation of AKT/mTOR, via the overexpression of *miR-29a*, thus controlling cancer cell proliferation in hepatocellular carcinoma (HCC). *MiR-29a* was claimed to have the ability to decreased proliferation in non-small-cell lung cancer (NSCLC), via negatively correlating with LIM and SH3 domain protein 1 (LASP1), a cAMP- and cGMP-dependent signaling protein and a member of the nebulin family of actin-binding proteins [50]. At the same time, the suppression of proliferation caused by *miR-29a* was also affirmed by Li et al. [51] partly via targetting cell division control protein 42 homolog (CDC42) in NSCLC. In addition, Pei et al. [52] demonstrated that, in BCa cells, *miR-29a* could induce cell proliferation by directly targetting ten eleven translocation (TET) 1 (TET1). TET1 was a member of the TET family and able to alter 5-methylcytosine (5mC) to 5-hydroxymethylcytosine (5hmC), which could induce CpG island demethylation in specific gene promoter [53]. Nonetheless, the newest research acknowledged *miR-29a* remarkably weakened cell proliferation in MCF-7 cells, one BCa cells, partly through tumor necrosis factor (TNF) receptor (TNFR) associated factor 1 (TNFR1), the prime receptor that commanded TNF-α-induced cellular events [54]. The absolutely opposite standpoint might be worthy of further discovery Figures 1–5 and Tables 1–3.

**Figure 1:** *MiR-29a* targetted p42.3, CDK2, CDK4, CDK6, MUC1, QKI-6, SPARC, CDC42, TNFR1 and thus inhibited proliferation However, *miR-29a* could also induce proliferation though KDM5B, TET1, PPARγ, SREBP-1c, LASP1.

**Figure 2:** MCL-1, KDM5B, QKI-6, MMP2, TNFR1 are the five target genes of *miR-29a* and *miR-29a* inhibited their functions and promoted apoptosis On the other hand, *miR-29a* decreased apoptosis by refraining HSP60 and motivating HSP27, HSP40, HSP70, HSP90. Abbreviations: HSP, heat shock protein; MCL-1, myeloid cell leukemia 1; MMP2, matrix metalloproteinase 2.

**Figure 3:** VASH2 and VEGF, inhibited by *miR-29a*, acted in a stimulative role in angiogenesis But, HBP1 and PTEN, which were also restrained by *miR-29a*, lessened angiogenesis. Abbreviations: HBP1, HMG box-containing protein-1; PTEN, phosphatase and tensin homolog; VASH2, vasohibin 2; VEGF, vascular endothelial growth factor.

**Figure 4:** *MiR-29a* magnified drug resistance via targetting PREN/AKT/GSK3β and Wnt/β-catenin and reduced drug resistance by binding to MUC1

**Figure 5:** Up-regulated *miR-29a* targetted TET1, MCL-1, LASP1, ITGB1, TFEB, ATG9A, Robo1, PI3K/AKT, MMP2, CEACAM6, TRIM68, PGK-1, TRAF4, VEGF-A, LOXL2, CDC42 directly and inhibited the expression of them resulting in decreasing cell metastasis Additionally, *miR-29a* could enhance metastasis via HUR, PTEN, TTP, KLF4. Abbreviations: CEACAM6, carcinoembryonic antigen-related cell adhesion molecule 6; ITGB1, integrin β1; MCL-1, myeloid cell leukemia 1; MMP2, matrix metalloproteinase 2; PTEN, phosphatase and tensin homolog; Robo1, roundabout 1; TTP, tristetraprolin; VEGF, vascular endothelial growth factor.

**Table 1:** Target genes and dysregulation of *miR-29a* in proliferation, apoptosis, angiogenesis, and drug resistance

hsa-*miR-29a*	Diseases	Target genes	References	Participation
Down-regulated	PCa	*KDM5B*	Li et al. [41]	Proliferation
				Apoptosis
	GC	*p42.3*	Cui et al. [45]	Proliferation
		*CDK2*	Zhao et al. [46]	Proliferation
		*CDK4*		
		*CDK6*		
		*VEGF*	Zhang et al. [42]	Angiogenesis
	PDAC	*MUC1*	Trehoux et al. [47,48]	Proliferation
				Drug resistance
	Pancreatic cancer	*Wnt/β-catenin*	Cai et al. [65]	Drug resistance
	GSCs	*QKI-6*	Xi et al. [25]	Proliferation
				Apoptosis
	HCC	*SPARC*	Zhu et al. [49]	Proliferation
	NSCLC	*LASP1*	Hu et al. [50]	Proliferation
		*CDC42*	Li et al. [51]	Proliferation
	(ALK+)ALCL	*MCL-1*	Desjobert et al. [23]	Apoptosis
	BCa	*TNFR1*	Zhao et al. [54]	Proliferation
				Apoptosis
	OSCC	*MMP2*	Lu et al. [24]	Apoptosis
	Glioma	*VASH2*	Jia et al. [58]	Angiogenesis
	OS	*TUT1*	Zhu et al. [44]	Proliferation
Up-regulated	BCa	*TET1*	Pei et al. [52]	Proliferation
		*HSPs*	Choghaei et al. [56]	Apoptosis

Abbreviations: ALCL, anaplastic large cell lymphoma; HSP, heat shock protein; MCL-1, myeloid cell leukemia 1; MMP2, matrix metalloproteinase 2; VASH2, vasohibin 2; VEGF, vascular endothelial growth factor.

**Table 2:** Target genes and dysregulation of *miR-29a* in metastasis

hsa-*miR-29a*	Dieases	Target genes	Reference
Down-regulated	PCa	*TRIM68*	Li et al. [76]
		*PGK-1*	
		*TRAF4*	Ahmed et al. [19]
		*BMP*	
		*MCL-1*	Pasqualini et al. [77]
	GC	*VEGF-A*	Chen et al. [78]
		*ITGB1*	He et al. [80]
		*hTERT*	
		*Robo1*	Liu et al. [82]
	HNSCC	*LOXL2*	Fukumoto et al. [98]
	lung adenocarcinoma	*CEACAM6*	Han et al. [79]
	NSCLC	*LASP1*	Hu et al. [50]
		*CDC42*	Li et al. [51]
	PDAC	*TFEB*	Kwon et al. [67]
		*ATG9A*	
	BCa	*Robo1*	Li et al. [81]
	OSCC	*MMP2*	Lu et al. [24]
	PTC	*PI3K/AKT*	Li et al. [83]
	Cholangiocarcinoma	*HDAC4*	Wang et al. [75]
	Glioma	*HSP47*	Zhao et al. [84]
Up-regulated	BCa	*TTP*	Gebeshuber et al. [71]
		*TTP*	Al-Ahmadi et al. [73]
		*HUR*	
		*TET1*	Pei et al. [52]
	Metastatic hepatoma cell	*PTEN*	Kong et al. [72]
	CRC	*KLF4/MMP2/E-cad*	Tang et al. [74]

Abbreviations: BMP, bone morphogenetic protein; CEACAM6, carcinoembryonic antigen-related cell adhesion molecule 6; HNSCC, head and neck squamous cell carcinoma; HSP, heat shock protein; ITGB1, integrin β1; MMP2, matrix metalloproteinase 2; PTC, papillary thyroid carcinoma; PTEN, phosphatase and tensin homolog; Robo1, roundabout 1; TTP, tristetraprolin; VEGF, vascular endothelial growth factor.

**Table 3:** The role of *miR-29a* in the diagnosis, treatment, and stages of carcinoma

*MiR-29a*	Tumors	Proliferation	Apoptosis	Angiogenesis	Drug resistance	Metastasis
Down-regulated	PCa	+	-	-	-	+
	GC	+	-	+	-	+
	PDAC	+	-	-	-	+
	Pancreatic cancer	-	-	-	+	-
	GSCs	+	-	-	-	-
	HCC	+	-	-	-	-
	NSCLC	+	-	-	-	+
	(ALK+)ALCL	-	+	-	-	-
	OSCC	-	+	-	-	+
	Glioma	-	-	+	-	+
	OS	+	-	-	-	-
	HNSCC	-	-	-	-	+
	BCa	-	-	-	-	+
	PTC	-	-	-	-	+
	Cholangiocarcinoma	-	-	-	-	+
	Lung adenocarcinoma	-	-	-	-	+
Up-regulated	BCa	+	+	-	-	+
	Metastatic hepatoma cell	-	-	-	-	+
	CRC	-	-	-	-	+

Abbreviations: ALCL, anaplastic large cell lymphoma; HNSCC, head and neck squamous cell carcinoma; PTC, papillary thyroid carcinoma.

### *MiR-29a* in cell apoptosis

Apoptosis was recognized as a highly regulated and controlled process of cell death that occurred in multicellular organisms. It was activated through two pathways, including the intrinsic pathway and the extrinsic pathway, both of which induced cell death by activating caspases, such as proteases or enzymes that degraded proteins [55]. An increasing number of researches had demonstrated that *miR-29a* played a significant role in promoting apoptosis via targetting several relevant effectors in human cancer. Desjobert et al. [23] claimed that the expression of *miR-29a* was critically decreased by an active NPM-ALK kinase in ALK-positive (ALK+) ALCL cells, partly through methylation regulation. And this kind of modulation played a fundamental role in the high expression of myeloid cell leukemia 1 (MCL-1). MCL-1, a major anti-apoptotic BCL-2 family member localized to the mitochondrial membrane of ALK+ ALCL cell, acted as a promotor in tumor cell survival through suppressing apoptosis. Moreover, *miR-29a* in PCa cell lines (PC-3 and LNCaP cells) induced apoptosis by affecting the methylation status of H3K4 through restraining the expression of KDM5B, which was mentioned elsewhere [41]. *MiR-29a* also largely inhibited the anti-apoptotic ability of OSCC cell via directly targetting matrix metalloproteinase 2 (*MMP2*) gene, thus negatively regulating the expression of MMP2, a well-known oncogenic gene [24]. The apoptosis of GSCs was promoted by *miR-29a* via targetting QKI-6, and the detailed pathway had been mentioned earlier [25]. Similarly, in BCa cells, *miR-29a* showed a great potential in inducing apoptosis partly though targetting TNRF1 [54]. However, Choghaei et al. [56] found that the absence of *miR-29a* promoted apoptosis in breast carcinoma through modulating members of heat shock proteins (HSPs), such as up-regulating HSP60 level and down-regulating HSP27, HSP40, HSP70, and HSP90 levels.

### *MiR-29a* in angiogenesis

Angiogenesis was generally accepted as a consequential characteristic of varied malignant neoplasm, which was a complex process modulated by a sequential pro-angiogenic and anti-angiogenic factors [57]. Generous researches illustrated that *miR-29a* might be relevant with angiogenesis in the development and progression of cancers.

Jia et al. [58] found that *miR-29a* functioned as a suppressor in the expression of vasohibin 2 (VASH2), via the knockdown of H19, one of the long non-coding RNAs (lncRNAs). VASH2 was normally accepted as an angiogenic factor, which could adjust the angiogenesis in glioma. Except VASH2, *miR-29a* apparently repressed the expression and secretion of vascular endothelial growth factor (VEGF), one of the most common proteins liberated from cancer cells that could promote angiogenesis in GC cells [42]. Nevertheless, it was revealed by Wang et al. [59] that *miR-29a*, modulated by TGF-β in a Smad4-dependent way, served as a promoter in angiogenesis, since *miR-29a* stimulated the AKT signaling in endothelial cells, by targetting phosphatase and tensin homolog (PTEN). Furthermore, *miR-29a*, mediated by HMG box-containing protein-1 (HBP1), might regulate the angiogenic properties of human endothelial cells [60]. HBP1, a tumor suppressor protein, was recognized to inhibite Wnt signaling and modulate cell proliferation in BCa cells [61]. As a result, it still remained to explore whether *miR-29a* functioned as a suppressor or an enhancer in the angiogenesis of tumors.

### *MiR-29a* in drug-resistance

Nowadays, in malignancy, mortality caused by chemotherapy resistance keeps increasing and Sin et al. [62] and Zhang and Yuan [63] speculated that miRNAs might be involved in the therapy of EGFR-tyrosine kinase inhibitors (EGFR-TKIs) resistance in NSCLC. Besides, agilent miRNA microarrays were carried out to examine the miRNA expression profiles of gefitinib-resistant human HCC827/GR-8-1 cell line and the parental HCC827 cell line. Interestingly, *miR-149-5p* was up-regulated in the gefitinib-resistant human HCC827/GR-8-1 cells and associated with acquired gefitinib resistance [64]. Based on the above researches, we learned that miRNAs had showed a great potential in the drug resistance of tumor and a daring hypothesis was made that *miR-29a* took a considerable part in the regulation of chemotherapy resistance.

Cai et al. [65] disclosed previously that *miR-29a* induced the resistance to gemcitabine (GEM) in pancreatic cancer cells, mediated significantly by the activation the Wnt/β-catenin signaling pathway. The Wnt/β-catenin signaling was widely recognized to participate in the chemotherapy resistance of a variety of malignant tumors such as HCC, head and neck tumor, and PCa [66]. Nevertheless, it was confused that Trehoux et al. [47] reported that *miR-29a* sensitized pancreatic cancer cells to GEM *in vitro* by targetting MUC1. Additionally, Kwon et al. [67] found that *miR-29a* sensitized chemotherapeutic resistant pancreatic cancer cells to GEM and increased cytotoxicity. Furthermore, *miR-29a* played an essential role in ADR resistance via inhibiting the PTEN/AKT/GSK3β pathway in BCa cell lines [68]. Zhong et al. [43] also proved that *miR-29a* was correlated with drug-resistant ADR and docetaxel (Doc), at least partly by targetting PTEN, which was generally acknowledged as a cancer-depressing gene, and it could also regulate kinds of cell processes, like growth, apoptosis, migration, and invasion [69]. Besides, *miR-29a* could enhance the chemosensitivity in OSCC, particularly*cis*-Diaminedichloroplatinum (CDDP) [24].

### *MiR-29a* in invasion and metastasis

Metastasis was the most important sequelae in the progression of cancer. Therefore, the mechanism of tumorigenesis and development were urgently needed for the prevention.

It was hypothesized in the ‘seed and soil’ for metastasis that migratory tumor cells leave the primary tumor via intravasation, disseminating throughout the body by the bloodstream, and eventually implantation in a distant organ. These consecutive steps require close interplay between miRNA and its various targets [70].

Initially, Gebeshuber et al. [71] detected that the up-regulation of *miR-29a* impaired the expression of tristetraprolin (TTP). TTP was recognized as a protein that was relevant with EMT and negatively modulated AU-rich elements (AREs) containing targets, such as tumor interleukin (IL)-3, IL-8, cyclooxygenase 2 (Cox2), VEGF, c-Myc, cyclin D1, and TNF-a, known as the promotors of tumorigenesis. As a result, the high expression of miR-29a induced invasion and metastasis of tumor in co-operation with oncogenic Ras signaling in human BCa. Moreover, it was also clarified by Kong et al. [72] that *miR-29a* promoted migration of hepatoma cell mediated by hepatitis B virus X protein (HBx), as it directly inhibited the expression of PTEN and thus regulated Akt phosphorylation. MiR-29a was concerned with the aberrant TTP-HuR axis and promoted the invasiveness of BCa cells [73]. Pei et al. [52] presumed the overexpressed *miR-29a* facilitated cell growth and migration through down-regulating TET1. And it was discovered by Lu et al. [24] that the enhanced ability to invade and metastasize resulted partly from the excessive expression of *miR-29a* by directly targetting *MMP2* gene in OSCC. Tang et al. [74] also claimed that *miR-29a*/MMP2 signaling pathway largely contributed to the invasion and metastasis of CRC. They found that *miR-29a* promoted CRC metastasis through modulating KLF4/MMP2/E-cad. In addition, *miR-29a* took a great part in the TGF-β1/miR-29a/HDAC4 pathway, which promoted metastasis of cholangiocarcinoma [75]. It was unbelievable that others found *miR-29a* could also serve as a completely adverse role in the metastasis of tumors. For example Li et al. [76] announced that the up-regulation of *miR-29a*, mediated by isoflavone inhibited cell growth and invasion. Because of its ability to down-regulate its target genes TRIM68 and PGK-1 in PCa, Ahmed et al. [19] elucidated in 2013 that the up-regulation of *miR-29a* decreased the expression of the TRAF4. TRAF4 was positively related with the expression of bone morphogenetic proteins (BMPs), which belong to converting growth factor-β (TGF-β) superfamily and are well known to take a grave part in the bone metastasis of PCa. Accordingly, *miR-29a* might produce a marked effect on the bone metastasis of PCa through decreasing the expression of BMP, via targetting TRAF4. At the same time, there was also a pathway about c-Myc, Hedgehog, NF-κB/*miR-29a*/TRAF4 in promoting the invasion and metastasis of PCa, as *miR-29a* was inhibited by c-Myc, which was overexpressed in PCa. Also, *miR-29a* diminished cell migration partly by directly targetting MCL1 in PCa [77]. *MiR-29a* functioned as an inhibition role in NSCLC via negatively modulating expression of LASP1 [50] and CDC42 [51], LASP1 functioned as a cAMP- and cGMP-dependent signaling protein and CDC42 was a protein involved in the adjustment of the cell cycle. *MiR-29a*, directly under-regulating VEGF-A, was identified to inhibit the tumor microvessel density, and then suppressing the invasion and metastasis of GC cells [78]. *MiR-29a*, accompanied with other tumor-suppressive miRNAs, such as *miR-26a/b, miR-29b/c*, and *miR-218*, apparently inhibited the migration and invasion of head and neck squamous cell carcinoma (HNSCC), via directly up-regulating LOXL2 [98]. *MiR-29a*, through targetting carcinoembryonic antigen-related cell adhesion molecule 6 (CEACAM6), also inhibited the metastatic behavior of lung adenocarcinoma cells, as CEACAM6 was involved in the adhesion, migration, invasion, and metastasis of tumor cells by integrin receptors [79]. Wound healing and transwell assays conducted by Zhao et al. [46] revealed that *miR-29a* decreased the metastasis of GC. He et al. [80] further explored that the expression of *miR-29a*, inhibited by the up-regulation of hTERT, enhanced the expression of integrin β1 (ITGB1) in GC cells, thus leading to the augmented invasive capacity of GC cells. On the other side, restoration of *miR-29a* restrained the expression of ITGB1 and inhibited GC cell metastasis [80]. *MiR-29a* reduced the migration and invasion of PDAC cancer cell by the way of blocking autophagy flux, as indicated by an augmentation of autophagosomes and autophagy markers, p62 and LC3B, a reduction in autophagosome-lysosome fusion, as well as the decreased expression of autophagy proteins, TFEB and ATG9A, which are critical for autophagy [67]. The role of *miR-29a* in inhibiting the metastasis of BCa, at least in part, lied in its negative regulation of Roundabout 1 (Robo1) in MCF-7 BCa cells, through both the expression of *Robo1* mRNA and protein [81]. Similarly, Liu et al. [82] acknowledged, in the same year, the same signaling pathway as Li et al. [81] in GC. The up-regulation of *miR-29a* obviously decreased AKT3 expression, via directly binding to the 3′-UTR of AKT3, thereby suppressing PI3K/AKT pathway activation, which were involved in multiple cellular functions in papillary thyroid carcinoma (PTC) [83]. *MiR-29a* refrained from glioma tumor growth and invasion through decreasing the expression of HSP47, also known as SERPINH1. HSP47 was a product of *CBP2* gene, located at chromosome 11q13.5, a region frequently amplified in human cancers [84].

### *MiR-29a* in potential clinical application

In clinical application, a desirable biomarker that could facilitate disease detection, stages, and prediction of outcome, and provided appropriate treatment for kinds of cancers. There was emerging evidence for the prognostic role of various miRNAs in cancers. Luckily, the abnormality of *miR-29a* had been found in several types of tumors and might provide novel cancer biomarkers. Exempli gratia, the level of *miR-29a* in serum was significantly correlated with the clinical stage [85]. And the serum levels of *miR-29a* were obviously higher in stage III CRC, compared with levels in the healthy individuals [27]. In stage II CRC, high expression of *miR-29a* was associated with a longer disease-free survival (DFS) [86]. Additionally, higher *miR-29a* levels were significantly related to longer overall survival in metastatic high-grade serous carcinoma [87]. On the other hand, *miR-29a* was also lower in the early-recurrence patients, compared with levels in non-early recurrence group [4], and the same in feces from CRC patients, compared with those from normality [88]. Meta-analysis of 281 CRC patients and 299 healthy controls [89] revealed that *miR-29a* may be a novel potential biomarker for CRC diagnosis.

## Discussion and conclusion

In this review, we focussed on the function of *miR-29a* in the progression of cancers, such as PCa, BCa, lung cancer, GC, PDAC, GSCs, HCC, OSCC, glioma, and so on. Consequently, it regulated a variety of biological processes, including proliferation, apoptosis, angiogenesis, invasion, metastasis, and drug resistance. In opposite, *miR-29a* was discovered to be oncogenically neutral in the pancreatic acinar carcinoma by Dooley et al. [90], no matter the development, nor the growth of pancreatic tumor. In particularly, *miR-29a* exhibited its tissue specificity in BCa, as its up-regulation in the progression of proliferation and metastasis. This phenomenon was quite different from that in other malignant tissue. Commonly, *miR-29a* was down-regulated in kinds of cancers regardless of proliferation, apoptosis, drug resistance, and metastasis. The distinct tissue specificity deserved further researches and might disclose a brand new mechanism in the therapy of malignancy.

In detail, *miR-29a* was associated with various target genes, like CDK2, MMP2, Wnt/β-catenin, VEGF, and so on. MMP2, a type IV collagenase, is widely recognized to promote tumor metastasis by decreasing the basement membrane [91]. CDK2, a member of protein kinase family, significantly modulated abundant events of eukaryotic cell division cycle [92]. VEGF was known to take a great part in the progression and metastasis of cancers through inducing angiogenesis [93]. Thus it can be seen that *miR-29a* adjusted these biological and significant genes and participated in tumorigenesis. However the adjustment of miRNAs is a complex network, which means that an miRNA could regulate multiple target genes, meanwhile, a single gene could be influenced by a variety of miRNAs, including *miR-29a*.

With the development of the depth of the sequencing and the recognition of tumor development, miRNAs were confirmed the relationship with materials which had never caught our eyes, such as extracellular vesicles (EVs), circular RNA, lncRNAs, and autophagy. For example, cell-derived EVs, loaded with functional miRNAs were delivered to the therapeutic targets, which might provide a novel therapies for cancers [94]. In addition, circular RNA modulated the proliferation and invasion of tumors though targetting miRNAs, which provided a novel insight for cancer biology [95–97]. All these potential mechanisms optimized the function of miRNAs. However, no one claimed that *miR-29a* was involved in the above mechanism and whether there were some mysteries about the tumorigenesis and tumor development. We considered that the connection, amongst miRNAs, EVs, circular RNA, lncRNAs, and autophagy, was interesting and urged us for further exploration.

In conclusion, *miR-29a* participated in cell proliferation, differentiation, apoptosis, angiogenesis, tumorigenicity, metastasis, drug-resistance, and so on. Increasing researches were involved in the function of *miR-29a* and the new findings or mechanism might also be related with *miR-29a*. We suggested that *miR-29a* serve as a potential therapeutic target and promising biomarker in various tumors, in future *miR-29a* requires further exploration.

## Abbreviations

BCa: breast cancer
BMP: bone morphogenetic protein
CDC42: cell division control protein 42 homolog
CDK: cyclin-dependent kinase
CEACAM6: carcinoembryonic antigen-related cell adhesion molecule 6
CRC: colorectal cancer
EGFR: epidermal growth factor receptor
EMT: epithelial-to-mesenchymal transition
EV: extracellular vesicle
GC: gastric cancer
GEM: gemcitabine
GSC: glioblastoma stem cell
HBP1: HMG box-containing protein-1
HCC: hepatocellular carcinoma
HSP: heat shock protein
ITGB1: integrin β1
LASP1: LIM and SH3 domain protein 1
lncRNA: long non-coding RNA
MCL-1: myeloid cell leukemia 1
MUC1: mucin 1
MMP2: matrix metalloproteinase 2
NSCLC: non-small-cell lung cancer
OSCC: oral squamous carcinoma
PCa: prostate cancer
PDAC: pancreatic ductal adenocarcinoma
PI3K: phosphoinositide 3-kinase
PTEN: phosphatase and tensin homolog
QKI-6: quaking gene isoform 6
Robo1: roundabout 1
TET1: ten eleven translocation 1
TNF: tumor necrosis factor
TNFR: TNF receptor
TTP: tristetraprolin
VASH2: vasohibin 2
VEGF: vascular endothelial growth factor
